This article has been retracted.

# MicroRNA-137 Contributes to Dampened Tumorigenesis in Human Gastric Cancer by Targeting AKT2

**DOI:** 10.1371/journal.pone.0130124

**Published:** 2015-06-23

**Authors:** Liping Wu, Jingtao Chen, Chunsheng Ding, Shutang Wei, Yanhong Zhu, Wenyi Yang, Xiaoyang Zhang, Xuejv Wei, Dazheng Han

**Affiliations:** Department of Gastroenterology, First affiliated Hospital of Henan University, Kaifeng, Henan, China; Columbia University, UNITED STATES

## Abstract

MiRNAs play important roles in tumorigenesis. This study focused on exploring the effects and regulation mechanism of miRNA-137 on the biological behaviors of gastric cancer. Total RNA was extracted from tissues of 100 patients with gastric cancer and from four gastric cancer cell lines. Expression of miR-137 was detected by real-time PCR from 100 patients. The effects of miR-137 overexpression on gastric cancer cells’ proliferation, apoptosis, migration and invasion ability were investigated in vitro and in vivo. The target gene of miR-137 was predicted by Targetscan on line software, screened by dual luciferase reporter gene assay and demonstrated by western blot. As a result, the expression of miR-137 was significant reduced in gastric cancer cell line HGC-27, HGC-803, SGC-7901 and MKN-45 as well as in gastric cancer tissues compared with GES-1 cell or matched adjacent non-neoplastic tissues (*p*<0.001). The re-introduction of miR-137 into gastric cancer cells was able to inhibit cell proliferation, migration and invasion. The in vivo experiments demonstrated that the miR-137 overexpression can reduce the gastric cancer cell proliferation and metastasis. Bioinformatic and western blot analysis indicated that the miR-137 acted as tumor suppressor roles on gastric cancer cells through targeting AKT2 and further affecting the Bad and GSK-3β. In conclusion, the miR-137 which is frequently down-regulated in gastric cancer is potentially involved in gastric cancer tumorigenesis and metastasis by regulating AKT2 related signal pathways.

## Introduction

Gastric cancer (GC) is the second frequent cause of death from cancer in the world [1]. So far, the mechanism of gastric carcinogenesis is largely unknown. The researchers have tried to study GC from the view of biochemistry and molecular biology that some tumor suppressor genes and tumor-related genes have been reported in GC. MicroRNAs (miRNAs) are endogenously small non-coding RNAs of 18~22 nucleotides that have been identified as posttranscriptional regulators of gene expression [2, 3]. MiRNAs play critical roles in lots of biological processes such as proliferation, development, differentiation, and apoptosis. Meanwhile, miRNAs have been validated to act as oncogenes or tumor suppressor genes during tumorigenesis. For example, miR-31 was identified as an oncogene in esophageal squamous cell carcinoma [4] and miR-451 functions as a tumor suppressor in human non-small cell lung cancer [5]. There are also many microRNAs were identified related to gastric cancer happening and development [6–13]. It has also been reported that the over-expression of miR-1, miR-20a, miR-27a, miR-34a and miR-423-5p can be used as diagnostic criteria of gastric cancer [14].Therefore, miRNAs are potential candidates of novel diagnostic biomarkers or therapeutic targets of gastric cancer.

MicroRNA-137 (miR-137) has been reported to be down-regulated and play roles as a tumor suppressor in colorectal cancer and oral cancer [15, 16]. However, the function of miR-137 and its mechanism underlying gastric carcinogenesis are still not very clear. Chen et al revealed that the miR-137 may plays as a tumor suppressor by targeting CDC42 to regulate cell cycle in gastric cancer [17]. Even so, it is clearly to us that the microRNA regulates biological behaviors by multiple path way that there could be more regulation mechanism of miR-137 toward GC tumorigenesis. In this study, we measured the expression of miR-137 in 100 patients with gastric cancer and investigated the roles of miR-137 in gastric cancer cells. We found some other functions of miR-137 in GC as well as another path way by which miR-137 played a role of tumor suppressor in GC tumorigenesis.

## Materials and Methods

### Ethics statement

All human studies have been approved by the appropriate ethics committee and have therefore been performed in accordance with the ethical standards. All persons gave their informed consent prior to their inclusion in the study.

### Patients and specimens

Human gastric cancer samples were collected from surgical specimens from 100 patients (male 56, female 44) with GC at the Cancer Institute and Hospital, First affiliated hospital of Henan University; the Second Hospital of the People's Liberation Army of China; Hebei Cancer Hospital. Non-tumor samples from the macroscopic tumor margin were isolated at the same time and used as the matched adjacent non-neoplastic tissues. All samples were divided into two parts. Tissue samples were collected immediately snap frozen in liquid nitrogen, and stored at -80°C until RNA extraction. The use of the tissue samples for all experiments was approved by the ethical board of the Institute of Basic Medical Sciences, Chinese Academy of Medical Sciences. All participants provided their verbal informed consent to participate in this study, and their verbal informed consents were written down. This onsent process was also approved by the ethics board. Four gastric cancer cell lines (HGC-27, SGC-7901, SGC-7901 and MKN-45) were all preserved in our laboratory and maintained in DMEM or 1640 with 10% FBS.

### RNA extraction, cDNA synthesis, and real-time PCR assays

Total RNA from tissues and cells was extracted by Trizol method (Ambion, USA) completely following the instructions. Single strand cDNA was synthesized by M-MLV (Ambion, USA) using 2 μg of total RNA as template. Oligo (dT)18 was used for mRNA reverse transcription while stem loop used for miRNA. Real time-PCR (RT-PCR) was performed by Bio-rad CFX96 (Bio-rad, USA) using SYBR mix (Tiangen, China). The PCR condition was: 95°C × 30s, followed by 40 cycles of 95°C× 5s, 60°C × 34s. For mRNAs, GAPDH was used as normalized control. For miRNAs, U6 snRNA was used for miRNA control. The relative expression of miR-137 was computed by 2-ΔΔCT method. Primer sequences are shown in Table 1.

**Table 1:** Primers used in this study.

Primers	Sequences (From 5’ to 3’)
GAPDH-F	TCAACGACCACTTTGTCAAGCTCAGCT
GAPDH-R	GGTGGTCCAGGGGTCTTACT
U6-F	CTCGCTTCGGCAGCACATATACT
U6-R	ACGCTTCACGAATTTGCGTGTC
U6-RT	AAAATATGGAACGCTTCACGAATTTG
miR-137-F	GCGCGC TTATTGCTTAAGAATAC
miR-137-R	GTGCAGGGTCCGAGGT
miR-137-RT	GTCGTATCCAGTGCAGGGTCCGAGGTATTCGCACTGGATACGACCTACGC
AKT2-F	GGTAGCCCAGAATGAGGA
AKT2-R	CAGGTGGCAGCATAAACA
AKT2_3’UTR_F	CTCCTGTACTAGCCGTTCC
AKT2_3’UTR_R	TACAGATGGATAGCTAGTTTATTAC
AKT2_M_F	TCGTGGTAAATGAGTACTCAAGG
AKT2_M_R	ACCACGAGATTACCTCTCTGCAA

### Plasmid construction

The miR-137 precursor sequence generated by annealing and miR-137-precursor-F and miR-137-precursor-R extension was meanwhile digested by BamHI and BglII, the products of which was inserts into the BamHI-BglII fragment of the pcDNA-GW/EmGFP-miR vector (GenePharma, China). At the meantime, negative control was also constructed.

### Cell culture and miRNA transfection

The cell lines HGC-27, SGC-7901 MKN-45 and GES-1 was purchased from the Cell Resource Center of Institute of Basic Medical Sciences, Chinese Academy of Medical Sciences and Peking Union Medical College (Beijing, China). The human gastric cell lines HGC-27, SGC-7901 and MKN-45 were cultured in RPMI 1640 (Gibco, BRL, UK) media supplemented with 10% fetal bovine serum and human gastric epithelium cell line GES-1 was maintained in DMEM (Gibco, BRL, UK) media. The miR-137 mimic and the scramble mimic which is non-homologous to the human genome were synthesized by GenePharma (Shanghai, China) and transfected into the cells to a final oligonucleotide concentration of 10nmol/L. All cell transfections were introduced by DharmaFECT1 Reagent (Dharmacon, TX, USA) according to the manufacturer’s used instructions. For each cell transfection two or three replication experiments were performed.

### Cell proliferation and apoptosis assay

Cell proliferation assay was performed by CCK8 method (DOJINDO, Japan). Briefly, the about 5000 miR-137 mimic transfected cells and scramble cells were respectively seeded into 96-well plates and cultured. Proliferation rates were determined at 0, 12, 24, 48, 72, 96 hours after transfection by adding 10µl CCK8 regent and tested according to the manuscripts. The apoptosis assays were tested in HGC-27 and SGC-7901 cells lines with or without miR-137 overexpression by Apoptosis Detection kit I (BD Biosciences, USA) and C6 Flow Cytometer (USA).

### Cell migration and invasion assays

We performed the wound-healing assay to test cell migration ability with or without miR-137 transfection. The artificial wounds were produced on the confluent cell monolayer with FBS free, using a 200 μL pipette tip at 24 hours post miR-137 transfection. The images were respectively taken at 0, 12, 24 and 36 hours after wound creation.

We then performed transwell assays to evaluate cells’ invasion ability. 5×10^4^ cells suspended in 200 μl medium without FBS were placed on the upper chamber of each insert with 430μl of 1 mg/ml matrigel (Millipore, USA). 600μl medium with 10% FBS as the nutritional attractant was put in the lower chamber. After 24 hours, the cells attached to the lower surface of chamber were ﬁxed 20 min by 20% methanol and stained for 10 min with 10% maygruwald-giemsa (MGG). The invasion membranes were then cut down and embedded under cover slips. We counted the cells in 3 different vision ﬁelds in condition with 20×magniﬁcation which were then used as the average number of cells. All assays were performed in three independent experiments.

### Animal experiment

The experiments involving animals were performed according to the Guide for the Care and Use of Laboratory Animals and the institutional ethical guidelines for animal experiments. The protocol was approved by the Committee on the Ethics of Animal Experiments of the CAMS (Chinese Academy of Medical Sciences) (Permit Number: C72-14-0664). All surgery was performed under sodium pentobarbital anesthesia, and all efforts were made to minimize suffering. Scramble-transfected and miR-137 overexpression HGC-27 cells (5 × 10^6^ cells) were inoculated s.c. into the dorsal flanks of BALB/c nude mice (female, Nu/Nu, 6 weeks old), all of which were purchased from the Animal Centre of Henan University and raised in pathogen-free conditions. The volume of tumor was measured for 5 weeks. All mice were killed and s.c. tumors were resected and the weight of tumors was tested. For in vivo metastasis experiments, HGC-27 cells were collected 24 hours after transfection. The cell viability assay was performed using an XTT assay kit24 hour post transfection according to the manufacturer's instructions (Roche, Tokyo, Japan). Then the mice (female, Nu/Nu, 6 weeks old) were injected with HGC-27 cells with or without miR-137 overexpression through the tail vein with 2×10^5^ cells in PBS. The HGC-27 cells were modified which can stably express luciferase (built by GENECHEM, Shanghai, China). The cells were checked by microscope to make sure that the cells were in good condition. After six weeks, Bioluminescence imaging was performed using an IVIS Spectrum and image radiance values were normalized using Living Image (Caliper Life Science, USA).

### Immunohistochemistry

Tissues were embedded into paraffin sections and treated 2 hours at 65°C and then deparaffinised. Before applying the primary antibodies at 4°C overnight, we carried out the antigen retrieval step. After that, slides were incubated with secondary antibody about 2 hours at 25°C conjugated to HRP (1:100; Zhongshanjinqiao, China). The Liquid DAB+ Substrate (zsgb-bio, China) was used for detection of the HRP activity.

### Luciferase miRNA target reporter assay

The full length of the 3’UTRs of human AKT2 mRNAs were each PCR amplified and cloned into the pMIR-REPORTTM Luciferase Reporter Vector (Ambion, USA) to generate the reporters. Mutations of the predicted seed regions in the mRNA sequences were created using primers including the mutated sites. HEK-293T cell were seeded onto 24-well plates (1 × 10^5^ cells per well) the day before transfections were performed. Cells (∼70% confluent) were transfected with pRL-TK luciferase reporters (50 ng/well), pGL-3firefly luciferase (10 ng/well), and mimic-137 (50 nmol/L, GenePharma, Shanghai, China) or scramble (50 nmol/L) using Lipofectamine 2000 (Invitrogen).Luciferase activities were measured using the Dual Luciferase Reporter Assay (Promega, USA).

### Western blotting

Proteins were separated on 10% SDS-PAGE and then transferred to 0.45 μm PVDF membranes (Amersham, UK). The membranes were incubated with 5% non-fat dried milk overnight at 4°C and with anti-AKT2 monoclonal antibody (Proteintech, USA) at 1:1000 dilution; anti-Bad monoclonal antibody (Bioworld, USA) at 1:500 dilution; anti-GSK-3B polyclonal antibody (Bioworld, USA) at 1:1000 dilution; anti-GAPDH antibody (Proteintech, Chicago, USA) at 1:30,000 dilution. After washing twice with TBST, the membranes were incubated with goat anti-rabbit antibody (zsgb-bio, China) at 1:5000 and 1:50000 dilutions for 2 h.

### Statistics

Each experiment was repeated at least three times. Student's t test (two-tailed) and the x^2^ test were performed, and statistically significant level was set at α = 0.05 two-side). Mean ± SD is displayed in the figures.

## Results

### MiR-137 is down-regulated in gastric cancer cells and clinical samples

We first examined the expression of mature miR-137 in 4 human gastric cancer cell lines (HGC-27, SGC-7901, SGC-7901 and MKN-45) and gastric epithelial cell (GES-1). These GC cell lines exhibited extraordinarily low expression of miR-137 compared to the GES-1 cell line (Fig 1A). To further study the relationship of miR-137 with GC occurrence, we detected the expression of miR-137 in 100 clinical patients (male 56, female 44; mean age 53 years) by Taqman probe-drived real-time PCR as described above. Out of 100 GC samples, the expression of miR-137 was down-regulated in 77 cases (77%) compared with adjacent tissues when the cut off was set up as 1.5. Meanwhile, miR-137 was up-regulated in 23 cases (23%) (Fig 1B and 1C). In general, the expression of miR-137 in GC tissues was lower than that in adjacent tissues in statistically significant differences (p = 0.00079, paired t-test, two-tailed, Fig 1C). Also, we have found a statistically significant association between the expression of miR-137 and gastric cancer clinical stage. The patients who have the lower levels of miR-137 expression were associated with high-grade and late-stage tumors (Fig 1D). These results indicated that alterations of miR-137 could be involved in gastric cancer progression.

**Fig 1:** MiR-137 expression in gastric cancer cells and clinical samples. **A.** MiR-137 expression ingastric cancer cell lines (HGC-27, SGC-7901, SGC-7901 and MKN-45) and gastric epithelial cell (GES-1). **B.** Four patients diagnosed as gastric cancer by H&E staining (original magnification, x100). **C/D.** MiR-137 expression in 100 clinical patients. **E.** Expression levelsof miR-137 in I–II stages (n = 38) versusIII–IV stages (n = 62) of the gastric cancer patients.

### MiR-137 inhibits cell proliferation in vitro and in vivo

We transfected miR-137 mimic into GC cell lines HGC-27 and SGC-7901, both of which showed great transfection efficiency (Fig 2A). The results of CCK8 growth assays at 0, 1, 2, 3 and 4 d after miR-137 and scramble transfection are shown in Fig 2B. Compared with scramble transfection, miR-137 transfection significantly reduced the proliferation of both cell lines (Fig 2B). Then we investigated the effect of miR-137 on cell apoptosis. The early apoptotic cells in the scramble group was about 10% in HGC-27 and 2.9% in SGC-7901, whereas after miR-137 transfection, the percentage of early apoptotic cells was increased to 17.5% in HGC-27 and 8.3% in SGC-7901, which showed significantly difference (Fig 2C). From these results, it can be concluded that miR-137 could suppress lung cancer cell survival by inducing early apoptosis.

**Fig 2:** Overexpression of miR-137 inhibits gastric cancer cell proliferation. **A.** Real-time PCR was performed to detect the miR-137 expression in HGC-27 and SGC-7901 cells treated with miR-137 mimic or scramble mimic. **B.** Growth of HGC-27 and SGC-7901 cells was shown after transfection with miR-137 mimic or scramble mimic or no transfection. The growth index was assessed at 0, 1, 2, 3 and 4 days. The bars represent the mean ± SD of three independent experiments (*** means *P*< 0.001). **C.** HGC-27and SGC-7901 cells were stained with PE Annexin V and 7-AAD 72 h after treatment with miR-137mimics or scramble. Early apoptotic cells are shown in the right quadrant. **D.** Representative figure of in vivo experiments. The tumor in miR-137 overexpression group is much smaller than the scramble. **E.** HE staining of mice tumor. **F/G.** Tumor volume and weight were calculated and all data are shown as mean ± SD. These results showed that both the tumor volume and weight was significantly reduced by miR-137 overexpression. These result verified that the miR-137 overexpression can suppress tumor growth in vivo (*: *p*<0.05;**: *p*<0.01; ***:*p*<0.001).

To further verify the findings above, an in vivo model was constructed. We found that tumor growth was significantly slower in the miR-137 overexpression mice than in the controls (Fig 2D, 2E and 2G). In agreement with the tumor growth curve, the weights of tumors induced by scramble cells were significantly higher than that by the miR-137 overexpression (Fig 2F). These results further confirmed that the miR-137 overexpression could limit the gastric cancer cell proliferation in vivo.

### MiR-137 inhibits cell migration and invasion in vitro and in vivo

We further assessed the effects of miR-137 on cell migration and invasion, which were the key determinants of malignant progression and metastasis. The effects of miR-137 on cell migration were demonstrated by a wound healing/scratch assay in HGC-27 and SGC-7901 cells. Both of two cell lines treated with miR-137 mimic were distinctively less migratory than scramble control or untreated cells at 12, 24, and 36 hours after scratching (Fig 3A). Furthermore, we conducted cell invasion assay to measure the directional invasion abilities of the cells after miR-137 overexpression. As a result, the invasiveness of cells transfected with miR-137 mimic was dramatically decreased compared with the scramble cells in HGC-27 and SGC-7901 (Fig 3B). Then, in vivo experiments were employed to further verify this result. We firstly demonstrated that cells transfected with miR-137 mimic or mimic control did not show a significant decrease in cell viability compared to untreated cells. Also, there is no difference in cell viability between the cells transfected with miR-137 mimic compared to negative control (S2 Fig). As shown in Fig 3C, the bioluminescent imaging of mice in the miR-137 overexpression group showed a much smaller image. Also, the number of lung metastasis per mice in miR-137 group showed a significantly lower level compared to scramble group, which indicated that the miR-137 could suppress metastasis in vivo. These results demonstrated that miR-137 played important roles in regulating cell migration and invasiveness in gastric cancer and suggested that the down-regulation of miR-137 might contribute to tumor metastasis in gastric carcinogenesis.

**Fig 3:** Overexpression of miR-137 inhibits gastric cancer cell migration and invasion. **A.** SGC-7901 and HGC-27 cells were not transfected or transfected with miR-137 mimics or scramble for 24 hours, and wounds were made. The relative ratio of wound closure per field is shown. As a result, cells transfected with miR-137 showed a significantly higher migrate speed compared to the control. **B.** HGC-27 and SGC-7901 cells were not transfected or transfected with miR-137 mimics or scramble for 24 hours, and transwell invasion assay was performed. The relative ratio of invasive cells per field is shown. Magnification for identification of migration is ×400 and invasion is ×40. This result demonstrated that the migration ability of lung cancer cells can be inhibited by miR-137 overexpression. **C.** Bioluminescentimaging (left) and the number of lung metastasis per mice (middle) showed that the miR-137 can suppress metastasis in vivo. The HE staining showed that the metastasis in mice lung (right).

### miR-137 targets AKT2 in GC

MiRNAs performed biological functions through negatively regulating their target genes. As predicted, there was complementarity between has-miR-137 and AKT2 3’-UTR (Fig 4A).

**Fig 4:** AKT2 is experimentally validated as a direct target of miR-137. **A.** Sequence of the miR-137 binding sites within the human AKT2 3’-UTR and a schematic diagram of the reporter constructs showing the entire AKT2 3’-UTR sequence (AKT2_WT) and the mutated AKT2 3’-UTR sequence (M1, M2). **B.** Luciferase activity of the AKT2_WT reporter and the AKT2_MUT reporter in the presence of 10 nmol/L of miR-137 mimic or scramble. **C.** Relative expression of AKT2 in HGC-27 and SGC-7901 cells not transfected or transfected with miR-137 mimics or scramble 24 hours. **D.** Immunoblotting of AKT2 in HGC-27 and SGC-7901 cells not transfected or transfected with miR-137 mimic or scramble. All data are shown as mean ± SD. **E.** Immunoblotting of Bad, GSK-3β, p-Bad and p-GSK-β.**f**Western blot analysis of AKT2 protein level in 12 GC patients in whom miR-137 was down regulatedin their GC tissues.

To test the hypothesis that AKT2 might be a target of miR-137, a reporter plasmid harboring the wild-type 3’-UTR region of AKT2 downstream of the luciferase coding region (Fig 4A, AKT2_WT) was constructed. HEK-293T cells were cotransfected with reporter plasmid (AKT2_WT) and scramble. As a result, miR-137 transfected cells showed a marked reduction (≈58%) of luciferase activity (Fig 4B). Then, the same assay was performed for another reporter plasmid containing mutated AKT2 3’-UTR in miR-137 binding sites. As expected, the inhibition of luciferase activity by miR-137 was partly removed with binding site 1 or binding cite 2 mutant and almost abolished in the AKT2_MUT double mutant, suggesting that the conserved region was fully responsible for miR-137 function (Fig 4B).

To further investigate the interaction between miR-137 and AKT2, HGC-27 and SGC-7901 cells were transfected with miR-137. AKT2 mRNA expression was determined by real-time PCR. No significant difference was observed between miR-137–treated and scramble-treated or untreated HGC-27 and SGC-7901 cells (Fig 4C). Then, western blotting analysis was conducted to measure the level of AKT2 protein. We found that the expression of AKT2 protein was down regulated in miR-137 treated HGC-27 and SGC-7901 cells, but not in scramble or untreated cells (Fig 4D). These data suggest that miR-137 directly recognizes the 3’-UTR of AKT2 mRNA and inhibits AKT2 translation. Thus, down regulated miR-137 in gastric cancer inhibits the suppression of AKT2, which in turn decelerate tumorigenesis.

AKT2 is a member of AKT family. We further detected its downstream effectors Bad and GSK-B. As a result, the p-Bad and p-GSK-B was obviously down regulated in miR-137 treated HGC-27 and SGC-7901 cells compared with scramble-treated or untreated cells. No significant change was found in non-phosphorylated Bad or GSK (Fig 4E). These findings suggest that the accelerated gastric cancer cell growth was partially due to the over-actived Akt pathways. Besides promoting cell proliferation, actived Akt could also phosphorylate Bad at Ser112 and Ser136, blocking Bad-induced cell death. In the absence of phosphorylation at these sites, Bad is thought to interact with Bcl-xl to induce cell death. In contrast, Akt-mediated hyperphosphorylation of Bad may promote cell survival in cancer cells. Our Western blotting results confirmed the above speculation that the change of gastric cancer cell activities in condition of miR-137-transfected cells could be a result of decreased phosphorylation of Bad. Furthermore, we analysed the protein levels of AKT2 in 12 GC patientsin whom miR-137 was down-regulated. Among these samples, AKT2 was up-regulated in9patientsin their GC tissues (Fig 4F).

### The restoration of AKT2 leaded to an activation of invasion and a suppression of apoptosis

In order to further demonstrate the roles of miR-137 and AKT2 played during tumorigenesis, we investigated the effect of restoration of AKT2 in miR-137 transfected cells. The western blot demonstrated that the AKT2 protein level in AKT2 overexpression sample was apparently higher than that of the negative control even under the suppression of miR-137. The restoration of AKT2 leaded to an activation of invasion and a suppression of apoptosis (Fig 5).

**Fig 5:** miR-137 active cell apoptosis and negatively regulate cell invasion by targeting AKT2. **A.** AKT2 protein level was assessed in GC cells treated by overexpression of miR-137 and/ or AKT2. **B.** AKT2 restoration leads to a suppression of apoptosis in GC cells while miR-137 promotes apoptosis. **C.** AKT2 restoration actives the apoptosis and invasion of GC cells while miR-137 showed opposite effects. Representative images are shown. The normalized ratio of invasive cells is shown in the bottom panels. In Fig 5, “miR-137” represents the cells transfected by miR-137 and pcDNA 3.1 empty vector. “AKT2_oe” represents the cells transfected by AKT2 overexpression vector. “miR-137 +AKT2_oe” represents the cells co-transfected by miR-137 and AKT2 overexpression vector. “Scr” represents the cells transfected with mimic negative control and pcDNA 3.1 empty vector.

## Discussion

miRNAs have been frequently indicated to be often dysregulated in diverse human cancers and some miRNAs has even been used employed as therapeutic targets of cancer. The researches referring to the relationship between miRNAs and cancers could help us with the understanding of cancer.

There are only a few researches referring the role miR-137 played in gastric cancer. It has been reported that the miR-137 is a negative regulator of Cdc42 and by targeting which inducing apoptosis and cell cycle G1 arrest in gastric cancer cells [17]. However, the regulation effect of microRNA in cancer is quite complicated. It seems impossible that the miR-137 regulates the gastric cancer by the single pathway. In this research, the function and mechanism that miR-137 regulated gastric cancer was further investigated.

Firstly, we detected the expression of miR-137 in 100 patients and found that the expression of miR-137 is significantly down-regulated in cancer sample. Also, we have found a statistically significant association between the expression of miR-137 and gastric cancer clinical stage. These results indicated that alterations of miR-137 could be involved in gastric cancer progression. We have tried to find the relationship between miR-137 and patients’ age and sex, but no statistic result was found. As the present study revealed that the expression of miR-137 was down-regulated in most of the GC tissues compared with adjacent tissues (77%), we could consider about the diagnosis and prognostic use of miR-137. Further validation in prospective studies is warranted and more accessible samples sources, such as miR-137–enriched tumor-derived exosomes from blood, should be investigated. Also, it should be noticed that to some extent the cut off value(cut off = 1.5) we chose could be still arbitrary. When it was set higher, there could be fewer patients with miR-137 down regulated in cancer tissues. However, even in this condition, there was about 23%of the cancers have high miR-137 expression. This may be due to the individual difference among patients that some of individuals may have different gene expression pattern during tumorigenesis or cancer progression.

As the expression of miR-137 in GC tissues was lower than that in adjacent tissues in statistically significant differences (p = 0.00079), we could speculate that this expression characteristic was associated with the cancer development. This speculation was confirmed by in vitro and in vivo studies that the miR-137 can negatively regulate the cell proliferation, migration and invasion. The miR-137 expression level can keep on a high level during a long period after transfection both in gastric cancer cell lines, end-stage xenograft tumors and inmetastatic location in lungs (S1A Fig–S1C Fig). However, the overexpression method leads to very high expression levels of miR-137 (Fig 2A). This high level of miR-137 may cause additional effects. For example, miR-137 is a negative regulator of Cdc42 and by targeting which inducing apoptosis and cell cycle G1 arrest in gastric cancer cells [17]. As the miR-137 in our study was upregulated thousands of times, it may lead to the inhibition of other targets such as Cdc42. Obviously, in this study we cannot exclude the possibility that the tumor suppressor effects of miR-137 was mediated by suppressing other target genes.

Then, we found that miR-137 acts as a tumor suppressor gene through targeting AKT2, which is a member of AKT family. The restoration of AKT2 causes the up regulation of AKT2 in miR-137 transfected cells, which is much higher than that in scramble. This may due to that the AKT2 overexpression reversed the protein level miR-137 suppressed. More importantly, the restoration of AKT2 regulates the apoptosis and invasion of gastric cancer cells, leading to an activation of invasion and a suppression of apoptosis (Fig 5). This rescue experiment provides further evidence that the miR-137 active cell apoptosis and negatively regulate cell invasion by targeting AKT2. In vivo experiments also demonstrated that the miR-137 expression is negatively relative to the AKT2 expression (S1D Fig and S1E Fig). AKT is a crucial factor of PI3K/AKT path way. The down regulation of AKT2 further affects its down-stream protein Bad and GSK-3B, that the p-Bad and p-GSK-B was obviously down regulated. Bad can play its’ roles by phosphorylation and further regulated the cell fate [18]. GSK-3B, which is also known as GSK-3β usually, controls the cell immigration and invasion. In conclusion, we have identified a link between miR-137 and AKT2 that is a novel constituent of gastric cancer tumorigenesis. The miR-137 has been demonstrated to be related to AKT2 regulation [19]. In hepatocellular carcinoma, miR-137 inhibits cancer cell growth and metastasis via directly targeting AKT2 [20]. In fact, we e have screened 8 genes as potential targets of miR-137 (S1 Table). However, the AKT2 is the only direct target of miR-137 after dual luciferase reporter gene assay and western blot investigation. From Fig 4D we can find thatmiR-137 can affect the AKT2 and p-AKT2in both HGC-27 and SGC-7901 cells. But interestingly, in SGC-7901 the phosphorylation status was apparently affected more. This phenomenon can be consistently observed in the three repeated blots we performed. We deducted that there could be due to the special property of different cancer cells. There might be specific regulation path way of miR-137 in SGC-7901 which repressed the phosphorylation status of AKT2.However, from the present research, we cannot fully explain this mechanism. When we chose the patients who have low expression of miR-137 in their GC tissue to detect the AKT2 protein expression, we found most of these patients(9/12) have high AKT2 level in their GC tissue. This result suggested that the miR-137 could target AKT2 in patients. There were also three patients who have low expression of AKT2 in GC tissue though the expression of miR-137 is low. This result may due to the individual difference among patients.

In conclusion, our expression and functional studies suggested that the miR-137 is frequently down-regulated in gastric cancer may act as a tumor suppressor in GC cells, reintroducing expression of which on GC cells suppressed gastric cancer cell proliferation, migration and invasion by directly targeting AKT2. Thus, our works is a good supplement to the previous work and is helpful for us to understand the miR-137 regulation mechanism in cancer.

## Supporting Information

S1 Fig miR-137 and AKT2 expression after transfection. A. miR-137 expression in HGC-27 cells and SGC-7901 cells 72 h post transfection. B. miR-137 expression in the end-stage xenograft tumors. C. miR-137 expression in metastatic localization of mice lungs. D. AKT2 expression in metastatic localization of mice lungs. We mixed the five lungs together in the same group. E. AKT2 expression in metastatic localization of mice lungs. We detected the Akt2 protein expression in each mouse respectively. 30 μg total protein was used for each sample.
(TIF)

S2 Fig Cell viability assay before metastasis experiment. Cell viability assay was performed 24 hours post transfection.
(TIF)

S3 Fig Adensitometric analysis of Fig 4E. (TIF)

S1 Table Potential target genes of miR-137. The potential target genes of miR-137 were predicted by on line software and detected by dual luciferase reporter gene assay and western bloting.
(DOCX)
